# Noncoding RNAs Act as Tumor-Derived Molecular Components in Inducing Premetastatic Niche Formation

**DOI:** 10.1155/2019/9258075

**Published:** 2019-06-12

**Authors:** Zhedong Zhang, Jiao Qiao, Dafang Zhang, Weihua Zhu, Jiye Zhu, Xisheng Leng, Shu Li

**Affiliations:** ^1^Department of Hepatobiliary Surgery, Peking University People's Hospital, Beijing, 100044, China; ^2^Department of Nephrology, Shandong Provincial Hospital Affiliated to Shandong University, Shandong, 250021, China

## Abstract

Cancer metastasis has been demonstrated as it is the culmination of a cascade of priming steps. Increasing evidence has shown that tumor-derived molecular components (TDMCs) are known as extra cellular vesicle and nonvesicle factors and serve as versatile intercellular communication vehicles which can mediate signaling in the tumor microenvironment while creating the premetastatic niche. Noncoding RNAs (ncRNAs) as one of the TDMCs have been proved in participating in the formation of the premetastatic niche. Understanding the premetastatic niche formation mechanisms through TDMCs, especially ncRNAs may open a new avenue for cancer metastasis therapeutic strategies. In this review, recent findings regarding ncRNAs function were summarized, and then the interaction with the premetastatic niche formation was studied, which highlight the potential of using ncRNAs for cancer diagnosis and therapeutic effect.

## 1. Introduction

Increasing tumor patients pass away eventually owing to tumor metastatic progression every year, even though significant advancements have been achieved in cancer therapies [1]. Therefore, it emphasizes the important goal of cancer research efforts to identify the pivotal molecular and cellular components in every step of tumor metastasis to develop new strategy for prevention and control of tumor metastasis. About 100 years ago, “seed and soil” hypothesis was originally proposed by Stephen Paget [2] which indicated that metastatic tumor cell “seed” chose the fertile “soil” to colonization. Under numerous efforts of research groups, it is now widely accepted that primary tumors prior modulate the local microenvironment of distant organs in preparation for tumor cell colonization even before their arrival. The microenvironment is termed the premetastatic niche with a series changes including immunosuppression, inflammation, lymphangiogenesis, organotropism, angiogenesis, and vascular permeability [3], which is crucial for the development of metastasis and has attracted more and more attention in the last several years [4].

TDMCs, one of the primary tumor-secreted molecules can be divided into nonvesicle tumor-derived secreted factors (TDSFs) and tumor-derived secreted extracellular vesicles (EVs) and carry diverse molecular components, such as proteins, lipids, RNA, and DNA molecules [5]. They have the functions of recruiting BMDCs, making the immune cells heterogeneity, altering the vasculature, and reprogramming the stromal cells and metabolic progress [6]. Studies have shown that ncRNAs are involved in regulating tumor transcription, invasion, and metastasis, etc., and may control cancer-related genes by acting on proteins [7].The expression of ncRNAs can be used to reflect the origin, grade, and other pathological constants of tumors and provide a method for the diagnosis and prognosis. In recent years, ncRNAs, as a new intercellular communication mechanism of TDMCs, have been established as an important part of premetastatic niche induction [8]. These new advances can indicate new direction to guide future research and better illustrate the potential mechanisms of tumor metastasis to design more effective diagnosis and treatment strategies to fight cancer. Here we focus on the most recent findings on the ncRNAs and their underlying induced mechanisms of the premetastatic niche formation.

## 2. NcRNAs as a Sort of TDMCs

In human genome sequence, only 2% of capacity is mRNA which can encode protein [9]. ncRNAs, known as nonmessenger refer to the RNAs without protein encoding function due to the lack of an open reading frame, and they are often transcribed from the complementary strand of protein encoding genes [10]. According to the length, ncRNAs are divided into long ncRNAs (lncRNAs) and short ncRNAs (< 200nt), and short ncRNAs include microRNAs (miRNAs) and PIWI-interacting RNAs (piRNAs). Based on the position, ncRNAs can be divided into nonvesicle and extracellular vesicle sort. With the development of extensively parallel sequencing technology and high-resolution microarrays, ncRNAs especially lncRNAs, miRNAs, and circRNAs have caught extended attentions. Massive lines of evidence suggested that ncRNAs are not only involved in life activities but also closely related to tumor cell differentiation, proliferation, migration, invasion, and infiltration [8, 11].

When ncRNAs function as one category of TDMCs, they mainly exist in the EVs and the minority of them are free [12]. EVs carry a distinctive repertoire of lncRNAs and short ncRNAs [13, 14]. What is more, packaging RNA into the EVs is also a selective progress [15]. EVs can transfer special sorts of RNAs from donor to recipient cells under pathological and physiological conditions [16] (Figure 1).

## 3. NcRNAs: A Key to the Formation of the Premetastatic Niche

Previous research has found primary tumor-derived vesicles contribute to the formation of the premetastatic niche [17]. Exosomes secreted by different cell types contain different RNAs and proteins that germinate from the primary tumor cells and enter the bloodstream, which may help the cancer change the metastatic microenvironment and invade new organs [18].

### 3.1. MiRNAs

Increasing angiogenesis and vascular permeability are essential for tumor development and metastasis, and tumor-derived EV miRNAs promote this progress by affecting endothelia cells [19, 20]. In the premetastasis niche, metastatic breast cancer cells secret EV-encapsulated miR-105 to destroy the vascular barriers by downregulating cellular endothelial tight junction protein zonula occludens 1 (ZO-1), which induces vascular leakiness in distant organs to promote metastasis [21]. Brain metastatic cancer cells-derived EVs of breast cancer contain miR-181c, which modulate the actin dynamics by the downregulation of phosphoinositide dependent kinase 1 (PDPK1) in brain endothelial cells to trigger blood brain barrier (BBB) destruction and facilitate cancer cells migration [22]. Distant lung fibroblast derived miR-30s stabilize pulmonary vessels in premetastatic lungs, the low expression of miR-30s could directly target the skp2 and promote pulmonary vascular destabilization via activating of matrix metalloproteinase 9 (MMP9) [23]. MiR-9, packaged in the SK23 melanoma cell-derived microvesicles (MVs) and delivered to the endothelial cells directly target the negative regulator suppressor of cytokine signaling 5 (SOCS5) and activating JAK-STAT signaling pathway to promote endothelial cell migration and tumor angiogenesis [24]. Exosomal miR-92a, derived from the leukemia cell line K562, has also shown the same function [19]. Exosomal miR-135b from chronic hypoxia multiple myeloma cells directly suppressed its target factor-inhibiting hypoxia inducible factor 1 (FIH-1) in endothelial cells and enhances the endothelial tube formation under hypoxia via the HIF-FIH signaling pathway [20]. Similarly, hypoxia can stimulate various miRNAs contain miR-210 overexpression in exosomes, so that promoting tumor angiogenesis [25].

The formation of premetastatic niche not only involves the angiogenesis and vascular permeability, but also the metabolic reprogramming and stromal reprogramming to facilitate tumor metastasis. Breast cancer can secret miR-122 enriched vesicles, which have been proved associated with breast cancer metastasis [26]. It can be taken up by the recipient premetastatic niche stromal cells such as astrocytes and lung fibroblasts to downregulate the glucose metabolism by decreasing the glycolytic enzyme pyruvate kinase (PKM) and glucose transporter 1 (GLUT1) [27]. Due to the availability of nutrient for the upcoming tumor cells, this new mechanism may be more important at an early stage prior to cancer-induced angiogenesis. What is more, EVs, rich in miR-494 and miR-542-3p, accelerate the premetastatic niche formation by targeting cadherin-17 and overexpressing the MMP2 and MMP3 in premetastatic lung stromal cells [28]. Transfection with a large amount of exosomal miRNAs (miR-100-5p, miR-21-5p, and miR-139-5p) in normal prostate fibroblasts increased the level of MMP2, MMP9, and MMP13 which relate to ECM and receptor activator of NF-*κ*B ligand expression [29]. Meanwhile, prostate cancer stem cells- (CSCs-) derived exosomes are different from bulk tumor derived in miRNA content which may modify the premetastatic niche by fibroblast migration and contribute to invasion [29]. In addition, exosomal miRNAs (miR-16, miR-21, and miR-29a) from tumor can bind to Toll-like receptors (TLR) in surrounding immune cells and trigger a TLR-mediated prometastatic inflammatory response [30]. Recently, a research shows that lung epithelial cells are critical for lung metastatic niche formation by tumor exosomal ncRNAs via TLR3 [31].

Therefore, most of the cancer-derived miRNAs, which packaged into vesicles as a class of small ncRNAs, to a certain extent play a crucial role in regulating numerous components and signaling pathway of premetastatic environment to facilitate metastasis. There is still spacious room for development in the function of various kinds of miRNAs in premetastatic niche formation.

### 3.2. LncRNAs

LncRNAs, such as CCAT2, DREH, HOTAIR, H19, lincROR, MALAT, and BCAR4, have relevant data and clinical significance in vivo and in vitro metastasis [32]. However, due to the less knowledge in the field, lncRNAs have been rarely studied in premetastatic niches.

With the increased studies of lncRNAs, they found that the imbalance of lncRNAs is involved in the regulation of tumor progression [33]. They can also release exosomes, change the cell physiology of remote nontumor cells, and enable the early survival of disseminated tumor cells in the premetastatic niche [34]. In CD90+ hepatocellular carcinoma cells, H19 is transferred and internalized by endothelial cells, and promotes angiogenesis and intercellular adhesion by upregulating the production and release of VEGF [35, 36]. Integrin *β*1/*α*5/JNK/c-JUN signaling pathway participates in higher matrix stiffness, which is induced LOXL2 increasing in liver cancer cells. LOXL2 promotes the production of fibrin, the expression of MMP9 and CXCL12, and the recruitment of BMDCs to help the formation of premetastatic niche [37]. In PDAC, exosome derived protein MIF can induce the formation of hepatic premetastatic niche and enhance the expression of liver metastatic. LncRNA Sox2ot regulate Sox2 expression to promote epithelial-mesenchymal transformation (EMT) and stem cell-like properties by competitively binding the miR-200 family [38]. Thereby, it promotes the invasion and metastasis of PDAC. The researchers from the University of Wisconsin School of medicine and public health hypothesized that anaplastic thyroid carcinoma (ATC) cancer stem-like cells (CSC) secrete lncRNAs transferred by exosome. It is important that linc-ROR induces EMT and establishes premetastatic niche [39] (Table 1).

### 3.3. CircRNAs

CircRNAs were once thought to be RNA splicing errors. However, they have now been shown to exist in many eukaryotic transcripts [40]. CircRNAs are mainly reported as miRNA sponges that affect downstream miRNAs target genes, regulate selective splicing, and affect host gene transcription [41]. Among circRNAs studies, miR-7 is the most studied miRNAs, which regulates multiple functions in the process of cancer, such as cell development, proliferation, and apoptosis [42].

The presence of circRNAs in exosomes was confirmed in cancer cell lines of hepatocellular carcinoma, colon cancer, lung cancer, gastric cancer, breast cancer, and cervical cancer. But circRNAs have not been reported in premetastatic niches.

### 3.4. Cross Talking

MiRNAs, LncRNAs, and circRNAs all have mutual regulation relationships, forming a cross talking network. NcRNAs and mRNAs can form a well-regulated interaction network [43]. It is well known that miRNAs play a role by targeting the 3 UTR of mRNAs [44]. LncRNAs-mRNAs interaction is like that of miRNAs-mRNAs. LncRNAs can bind to multiple mRNAs, and one mRNA can be targeted by multiple lncRNAs [45].

MD et al. summarized four ways of interaction between lncRNAs and miRNAs. The first is that LncRNAs are precursor molecules of miRNAs, for example, the precursor of H19 encoding miR-675 [46]. The second is that miRNAs reduce the stability of lncRNAs. Yoon et al. reported that RNA binding protein HuR recruits let-7/Ago2 to degrade lncRNA-p21 [47]. Thirdly, LncRNAs compete with miRNAs. For instance, the antisense transcript of CDR1 is almost completely complementary to miR-671 which can guide the degradation of the antisense transcript of CDR1 by AGO2-dependent methods [48]. Finally, as a sponge of miRNAs, LncRNA X chromosome inactivated specific transcript (XlST), inhibited the expression of miR-499a and promoted the expression of B-cell lymphoma-2 (Bel2) [49]. LncRNAs competitively bind to miRNAs as competitive endogenous RNA (ceRNA) [50].

CircRNAs have a sponge-isolating effect on miRNAs [51]. Cirs-7 (CDR1as) was found to isolate tumor suppressor miR-7 which inhibits EGF receptors in oncogenes such as IRS-1, IRS-2, and Raf1 in glioblastoma [52]. The ciRs-7/miR-7/miR-671 axis confirmed the significance of circRNAs entrapment on miRNA in cancer (Figure 2).

## 4. Clinical Utility of ncRNAs

### 4.1. TDMCs: A Source of Novel and Specific Biomarkers of Cancer

Early detection of reliable cancer biomarkers is critical to diagnosis. Ideally, biomarkers should be targeted to specific tumor types and detected noninvasive techniques prior to transfer. Tumor-derived exosomes are involved in the interstitial interaction between tumor cells and surrounding tissues and promote the development of malignant tumors.

Circulating miRNAs have great potential as a biomarkers. They bind to exosomes/microvesicles or protein complexes and are chemically stable to RNase activity and reproducible in the blood. Rodriguez M et al. confirmed that miR-196a-5p and miR-501-3p were downregulated in prostate cancer samples by rt-qPCR analysis in an independent cohort study, suggesting that specific miRNAs in urinary exosomes may serve as a noninvasive biomarker for the diagnosis of prostate cancer [53]. A higher level of circulating miR-122 was detected in early breast cancer metastasis progression [54], and a lower level of miR-125b in serum circulating exosomes of advanced melanoma could be used as a predictive marker [55]. In addition, these EVs can be used for the detection of tumor metastasis. The exosomes of patients with metastatic sporadic melanoma were compared with familial melanoma or the unaffected control group, and higher expression levels of miR-17, miR-19a, miR-21, miR-126, and miR-149 were found [56]. Exosome miR-21 is associated with esophageal cancer recurrence and distant metastasis [57]. Fleming et al. demonstrated that evaluating miR-15b, miR-30d, miR-150, and miR-425 was more likely to predict melanoma recurrence than TNM staging [58].

In addition to miRNAs, lncRNAs associated with tumor-derived exosomes are also attractive as potential biomarkers. LncRNA PCA3 (DD3) is an approved urinary biomarker and prebiopsy diagnosis of prostate cancer [59]. Elevated lncRNA ZFAS1 in serum exosomes of GC patients may represent a better biomarker for GC diagnosis [60]. In 2015, the plasma study of liver cancer patients found that lncRNA XLOC_014172 and LOC149086 are potential biomarkers for liver cancer metastasis [61]. Furthermore, the release of the regulation of high specific expression of lncRNAs in tumor tissues can be used as targets for the treatment of cancer [62].

CircRNAs, which are stably expressed in exosomes, are promising candidates for cancer biomarkers. Many circRNAs exhibit tissue-specific and developmental stage-specific patterns. CircRNAs are also described as biomarkers of aging in Drosophila [63]. In gastric cancer, the abundance of Hsa_circ_002059 was low. It was also lower in cancer tissues and adjacent tissues [64]. Chen et al. found that circPVT1 was upregulated in gastric cancer. It was an independent prognostic indicator for overall survival and disease-free survival of gastric cancer patients. This finding suggests that circPVT1 is a new prognostic marker for gastric cancer [65].

NcRNAs in circulating EVs may be a new and specific source of cancer biomarkers. Currently, the use of multiple circulating ncRNAs as reference genes may be more applicable.

### 4.2. Targeting ncRNAs in the Premetastatic Niche for Cancer Therapeutics

#### 4.2.1. The Therapeutic Potential of ncRNAs

NcRNAs have been proved to play an important role in tumorigenesis, typing, metastasis, drug resistance, and therapeutic effect [66]. Hence, many ncRNAs can be targeted for tumor therapy. What needs to be further investigated is how to consume EV or block the uptake of EV in cancer patients [67]. Functional studies have confirmed that miRNAs dysfunction is the cause of many cancers. MiRNA mimics and miRNA-targeting molecules (antimiRs) show promise in preclinical development [68]. MiRNAs have also been used in studies to sensitize tumor cells to chemotherapy. MiR-375 cotransports cisplatin nanoparticles as a promising treatment for liver cancer [69]. The fact that most lncRNAs are carcinogenic and upregulated during cancer suggests the possibility of therapeutic intervention. The specificity of lncRNAs has been used to selectively kill tumor cells, providing a pathway for targeted therapy. In addition, gene therapy can be tried to deliver beneficial tumor suppressor lncRNAs [70]. As for circRNAs, inhibiting the relevant f-circRNAs may be a new therapeutic approach, especially in the fight against cancer drug resistance [71].

#### 4.2.2. Therapeutic Target Groups of Specific ncRNAs

Before precise tumor treatment, it is very necessary to study the best miRNA candidates or miRNA targets for each disease. Recently, miR-CLIP seq technology can identify miRNA-mRNA association and sequencing [72]. The miR-CLIP capture technique can also identify the interaction between miRNAs and lncRNAs [73]. For example, the sponge effect of lncRNA H19 on mir106a upregulated the corresponding mRNA level [74]. In addition, it will be necessary to further understand the interaction between lncRNAs and circRNAs.

#### 4.2.3. Small Interfering RNA (siRNA) Therapy

To date, miRNAs and small interference RNAs (siRNA) play an important role through RNAi mechanism and are widely used in gene therapy, especially in cancer therapy. The efficiency of siRNA depends on a number of factors, such as targeted sequences, end modification, and whole-body delivery methods [75]. One of the most commonly used methods to inhibit the upregulation of carcinogenic lncRNAs is to deliver siRNA to target cells. Furthermore, lncRNAs expression was inhibited by the use of antisense oligonucleotide (ASO) or small molecule inhibitors [76]. Among them, some are undergoing Phase III clinical trials in prostate cancer, so far; however, most are still in the period of basic research [77].

#### 4.2.4. NcRNAs Replacement Therapy

One is the use of antimiRs, common inhibitors AntigomiRs, locked nucleic acid (LNA), etc., to block the expression of miRNAs targeting mRNA in tumor and premetastatic niche [78]. MiR-15a and miR-16-1 provide indications for miRNA-based treatment, and strong regulation of clonal amplification of CLL plays a role at the level of mature leukemia [79]. AntimiRs targeting miR-122 have reached phase II clinical trials for hepatitis [80]. MiR-10b antagomirs inhibit the metastasis of breast cancer in mice by silencing endogenous miR-10b, which is well tolerated in animals and is a promising candidate for the development of new antimetastatic drugs [81].

The second is the use of miRNAs mimics, which are a new therapeutic approach. In order to protect miRNAs from degradation by serum nucleases, miRNAs mimics were specifically delivered to tumor interested miRNAs by using the nanoparticle delivery system [82, 83]. For example, MiR-125b was directly injected into subcutaneous tumors using a nonviral vector composed of cationic polymer polyethylamine (PEI), targeting VE-cadherin to induce nonfunctional angiogenesis and inhibit tumor growth [84]. MiR-34, an analogue of tumor suppressor, has reached stage I clinical trials for the treatment of cancer [85]. Other ncRNAs have not been explored for their functional regulation.

AntimiRs drugs combined with chemotherapy or targeted therapeutic drugs (such as small molecules or antibodies) are used to reduce miRNAs, potential checkpoint inhibitors, and to reduce adverse reactions. Therefore, further studies are needed to resolve some controversial issues to achieve the clinical application of exosomes in the microenvironment of premetastatic niche.

## 5. Conclusions and Perspective

From traditional therapy to molecular targeted therapy, great progress has been made in the treatment of primary tumors. However, for the treatment of the formation of premetastatic niche, how to identify and kill the premetastatic niche at an early stage, and how to avoid the toxic and off-target effects of ncRNAs drugs targeted premetastatic niche need to be solved urgently.

As one of TDMCs, ncRNAs has been confirmed to be involved in the formation of premetastatic niche. By understanding the formation mechanism of premetastatic niche through TDMCs, especially ncRNAs, the hypothesis of premetastatic niche is further studied, which may provide new strategies for us to develop new targeted antitumor drugs, thus greatly improving the therapeutic effect and prognosis of tumors. In this regard, siRNA therapy and ncRNAs replacement therapy through exosomes are promising strategies with initial results, while the physiological and pathological effects of exosomes such as lncRNAs and circRNAs in the premetastatic niche still need to be further studied. Moreover, the latest miR-CLIP seq technology and miR-CLIP capture technology recognize the association between miRNAs and mRNAs, miRNAs and lncRNAs, respectively. The cross talking of miRNAs with circRNAs, lncRNAs, and circRNAs is for further study. In the future, identify the interactions between ncRNAs before performing precise tumor therapy, study the optimal ncRNA candidates or ncRNA targets for each disease, and target inhibitors for their interaction, which may provide the next generation of precise personalized drugs.

## Figures and Tables

**Figure 1:** The functions of ncRNAs. The molecular functions of lncRNAs can be summarized into decoy and miRNAs sponge and affect the stability of mRNAs by combining with mRNAs. And circRNAs competitively bind miRNAs as ceRNA.

**Figure 2:** Mechanism of premetastatic niche formation. Primary tumors prior modulate the premetastatic niche in preparation for tumor cell colonization even before their arrival. TDMCs have the functions of recruiting BMDCs, making the immune heterogeneity, altering the vasculature, and reprogramming. They create premetastatic niche as the signal transduction mediators. NcRNAs, one of TDMCs, are involved in the formation of premetastatic niche. MiRNAs, lncRNAs, and circRNAs are building a well-regulated interaction network by directly regulating with each other.

**Table 1:** Recently reported ncRNAs-mediated adaptations in a premetastatic niche.

ncRNAs species		Cancer type	Biological function	Mechanism	Refs
miRNA	miR-9	melanoma	promote migration and angiogenesis	target to SOCS5 and activating JAK-STAT signaling pathway	[24]
	miR-16, miR-21, miR-29a	lung cancer	promote tumor growth and metastasis	bind with TLR, trigger TLR-mediated pro-metastatic inflammatory response	[30]
	miR-92a	leukemia	regulate endothelial gene expression	Downregulate target gene integrin a5, play a similar role in endogenous miRNAs in HUVECs	[19]
	miR-100-5p, miR-21-5p, miR-139-5p	prostate cancer	modify pre-metastatic niche	increase MMP2, 9, 13, RANKL and fibroblast migration	[29]
	miR-105	breast cancer	promote metastasis	destroy the vascular barriers by downregulating ZO-1	[21]
	miR-122	breast cancer	induce angiogenesis	downregulate the glucose metabolism by decreasing PKM and GLUT1	[26]
	miR-135b	multiple myeloma	enhance endothelial tube formation under hypoxia	suppress FIH-1 in endothelial cells via the HIF-FIH signaling pathway	[20]
	miR-181c	brain-metastatic breast cancer	facilitate migration	downregulate PDPK1 in brain endothelial cells to trigger BBB destruction	[22]
	miR-210	leukemia	affect angiogenesis	exosomes containing a high expression level of miR-210 downregulate EFNA3	[25]
	miR-494, miR-542-3p	pancreatic adenocarcinoma	accelerate the pre-metastatic niche formation	target cdh-17 and over express MMP2 and MMP3	[28]
lncRNA	H19	hepatocellular carcinoma	promote angiogenesis and intercellular adhesion	up-regulate the VEGF, promote MMP9, CXCL12, and the recruitment of BMDCs	[35–37]
	LncRNA Sox2ot	Pancreatic duct adenocarcinoma	promote the invasion and metastasis	regulate Sox2 expression by binding the miR-200 family competitively	[38]
	lncRNA MALAT1, linc-ROR	anaplastic thyroid carcinoma	establish pre-metastatic niche	induce EMT	[39]
